# Glycine Improved Cryopreserved Spermatozoa Quality in Achai Bull

**DOI:** 10.1155/2022/8282387

**Published:** 2022-08-04

**Authors:** Muhammad Sohail Nazif, Zia ur Rehman, Humayun Khan, Farhan Anwar Khan, Tarique Hussain, Adnan Ahmad, Farmanullah, Ali Husnain, Safdar Muhammad, Ghulam Murtaza, Liu Gang

**Affiliations:** ^1^College of Veterinary Sciences, Faculty of Animal Husbandry and Veterinary Sciences, The University of Agriculture, Peshawar, Pakistan; ^2^Animal Sciences Division, Nuclear Institute for Agriculture and Biology (NIAB), Faisalabad 38000, Pakistan; ^3^Department of Animal Breeding and Genetics, Faculty of Veterinary and Animal Sciences, National Center for Livestock Breeding Genetics and Genomics, Lasbela University of Agriculture, Water and Marine Sciences, Uthal, Baluchistan, Pakistan; ^4^Key Laboratory of Agricultural Animal Genetics, Breeding and Reproduction, Education Ministry of China, College of Animal Sciences and Technology, Huazhong Agricultural, University, Wuhan 430070, China; ^5^Department of Animal Reproduction, Faculty of Animal Husbandry and Veterinary Sciences, Sindh Agriculture University, Tandojam, 70050 Sindh, Pakistan; ^6^College of Bioscience and Biotechnology, Hunan Agricultural University, Changsha, 410128 Hunan, China

## Abstract

Achai is a small size cattle breed, resilient to harsh and cold environment. Cryopreservation of Achai bull semen may help to improve its genetics and preserve the germplasm. Reactive oxygen species (ROS) affects the structural and functional integrity of the spermatozoa. During freezing and thawing processes, the ROS make changes in the spermatozoa quality parameters and reduce total antioxidant capacity (T-AOC) of semen that is considered as marker of oxidative stress. This study was designed to determine the effect of glycine along with vitamin E on post-thawed spermatozoa quality and total antioxidant capacity in Achai cattle. The semen collection was done twice a week from four mature fertile Achai cattle bulls (*n* = 4). The glycine was utilized as 0 mM, 5 mM, 10 mM, 15 mM, and 20 mM along with vitamin E @ 2.3 mM added constantly in each concentration. The control group contained all extenders except glycine. The results revealed that post-thawed spermatozoa motility was found significantly higher (*P* < 0.05) at 10 mM as compared to 5 mM, 15 mM, and 20 mM. Compared with control group, glycine concentration at 10 mM and other concentrations increased progressive and fast motility (%), curvilinear, straight line, and average path velocity (*μ*m/s). Moreover, beat cross frequency (Hz) was higher (*P* < 0.05), and post-thaw viability (%), plasma membrane integrity, and mitochondrial membrane potential were significantly higher (*P* < 0.05) at 10 mM of glycine concentration in comparison to control and other glycine concentrations. Besides, acrosome integrity (%) and DNA integrity (%) as well as post-thawed T-AOC were also significantly higher (*P* < 0.05) at 10 mM of glycine concentration as compared to other glycine concentrations and control group. It is concluded that 10 mM of glycine along with vitamin E @ 2.3 mM improved cryopreserved semen quality of Achai bull.

## 1. Introduction

Livestock is the main subsector of agriculture which contributes 58.92% to agriculture and 11.11% to the overall GDP. The milk, meat, and hides are the demands for sustainable livelihood. Pakistan is endowed with best breeds of the buffalo and cattle, and approximately, 96% milk is produced from these animals [1]. Among the cattle breeds, Achai cattle is one of the famous breeds found in northern areas of Hindu Kush Mountains [2]. It is reared under subsistence production system in hilly areas where scarcity of fodder is common. This breed has a dairy and light draught characteristic having disease resistance. It has better rearing capabilities than other cattle breeds and has low ration requirement. Due to the above-mentioned characteristics, this breed deserves more attention from local authorities. There is a dire need to have more research on Achai cattle to improve its health and reproductive performance [3].

Frozen semen helps to improve genetics, preserve endangered species, and easy transport of genetic material. Cryopreservation during semen preservation subjects the spermatozoa to acrosomal damage and other spermatozoa abnormalities and thus is associated with reduced post-thawed spermatozoa quality parameters. It has been estimated that 50% spermatozoa livability is dropped during semen cryopreservation due to different stressors, i.e., osmotic stress, oxidative stress, and cold shock. Semen extenders are being used since long to minimize these adverse effects on spermatozoa [4, 5].

Oxidant level is another factor that can affect semen quality. A limited concentration of oxidants is advantageous for spermatozoa's physiological functions. The production of free radicals is associated with the physiology of spermatozoa hyper-activation, capacitation, acrosomal reaction, and fertilization. Similarly, the production of reactive nitrogen species (RNS) is also formed resulting in increased level of these ROS and RNS that damage the spermatozoa due to oxidative stress [6, 7]. A 20% lowered fertilization rate has been reported in AI as compared to fresh semen owing to high level of ROS and RNS. Spermatozoa damage leads to higher rate of fertilization failure, abortion, and decreased fertility in males [8].

Inclusion of antioxidants results in improved post-thawed total motility of the spermatozoa and avoids damage using suitable level of semen extender for cattle [9]. Different antioxidants like carotenoids and flavonoids protect spermatozoa from harmful effects of cryopreservation and oxidation through co-enzymes and vitamins [10]. Furthermore, it is reported that antioxidants scavenge the free radicals and neutralize the production of ROS [11].

Glycine is an amino acid that plays a crucial role in preventing spermatozoa cell damage during cryofreezing and has been reported in goats and rams [12, 13]. Addition of glycine with glycerol in extender improved post-thaw spermatozoa quality. Several other studies have reported a positive effect on post-thaw semen quality in goats, after cryopreservation with glycine and other amino acids [14]. In addition, studies describe the inclusion of amino acids to semen extender that enhanced post-thawed spermatozoa motility, sustainability, acrosome integrity, and membrane integrity in buck, Zebu bulls [15], ram [16], stallion and donkey [17], and boar [18]. Vitamin E is a hydrophobic antioxidant that prevents peroxidation of phospholipids and protects spermatozoa cell membrane [19]. Further, the inclusion of vitamin E in semen extender may enhance semen quality through reduction of free radicals [20]. Comprehensive analysis is required for the assessment of various antioxidants from different sources in Achai bull semen. glycine and vitamin E have the potential to be used as antioxidants for the improvement of post-thaw spermatozoa quality of Achai bull semen. Current study was carried out to determine the antioxidant efficacy of glycine and vitamin E on the post-thawed spermatozoa quality in Achai bull semen.

## 2. Materials and Methods

### 2.1. Experimental Animals

The experimental approval was granted by the ethical committee of the Faculty of Animal Husbandry and Veterinary Sciences and semen processing unit, the University of Agriculture, Peshawar, Pakistan. Four fertile Achai cattle bulls, aged 4 to 6 years, having weight of 300-350 Kg, body condition score (BCS) 3-4, were selected with no provision of disease history. The semen was performed during summer season for a period of approximately six weeks. During that period, the temperature was around 35 to 40°C. The bulls were provided standard ration and *ad-libitum* fresh water. Green fodder was made available to all animals equally.

### 2.2. Collection and Processing of Semen

Semen samples were collected with artificial vagina having temperature 42°C twice a week. After collection, the ejaculates were incubated in water bath at 37°C until the volume, pH, concentration, and motility parameters were measured. Each ejaculate was examined with naked eyes in glass tube. Ejaculate having no contamination like blood or dirt was recommended for further processing. Each sample volume was recorded by using graduated collection tube. Mass activity was observed by putting an undiluted drop of semen on glass slide under warm stage of microscope and recorded as follows: 0 marked no mass motility, + marked as >20 percent of spermatozoa showing progressive motility, ++ marked as 40-60 percent showing progressive motility with slow wave, +++ marked as 60-80 percent showing progressive movement with wave more intense, and ++++ marked as 80 to 100 percent showing progressive movement with rapid wave waking eddies.

The samples met the minimum requirement (motility >65%) after initial evaluation of semen and then were pooled. The same spermatozoa motility was reported by others in previous studies using Achai cattle [21, 22]. The semen samples found with average pH 6.4 were measured by using digital pH meter, and the same pH was reported by others in previous studies [23, 24]. The pooled semen samples were assigned into five aliquots in water bath at 37°C. Different concentrations of glycine (Sigma Aldrich, USA), 0 mM, 5 mM, 10 mM, 15 mM, and 20 mM, were made and mixed directly into semen extender. Vitamin E @ 2.3 mM in each group of glycine was also added and mixed thoroughly, and the dose rate was selected in reference to the previous research [25]. The control group contained all extenders including vitamin E except glycine. The composition of semen extender is depicted in Table 1. Tris-based diluent was used for freezing of Achai bull semen. The pooled semen samples from four bulls were divided into five aliquots as mentioned above, and each aliquot was diluted with tris 3.07 g, citric acid 1.64 g, fructose 1.26 g, benzyl penicillin 1000 IU/mL, streptomycin sulfate 100 *μ*g/mL, glycerol 5%, and egg yolk 25%, and doubled-distilled water was added up to 100 mL. The spermatozoa concentration was kept twenty million (approximately) in 0.5-mL straw. The samples after dilution were incubated in cold cabinet at 4-5°C for 5-6 hours for equilibration. The straws were marked according to experimental design and filled by using automatic filling machine (IMV, France). Later on, the semen straws were kept for 10 minutes at 4 cm above the liquid nitrogen vapors. Thereafter, semen straws were dipped into liquid nitrogen (LN_2_) and were stored in LN_2_ container until further analysis. All the experiments were performed in triplicates. For motility, viability, plasma membrane integrity, acrosome integrity, DNA integrity, mitochondrial membrane potential, and T-AOC evaluation, five semen-filled straws were thawed for 20-30 seconds in water bath at 37°C. Mass motility was determined using a 20 *μ*L of undiluted semen on prewarmed slide at 37°C without using a coverslip and examined through (40×) phase contrast microscope (Olympus CX-41, Japan). Semen extender was prepared with little modification as described by (PARC/JICA) [26].

### 2.3. Post-Thaw Semen Evaluation

#### 2.3.1. Spermatozoa Motility Parameters, Velocity Distribution, and Kinematics

Thawing of frozen semen was done at 37°C for 20-30 seconds in a water bath and subjected to post-thaw evaluation following semen characteristics.

Spermatozoa kinematics was examined using computer-assisted semen analysis (CASA, AndroVision CASA system; Minitube, Germany). A total of 10 *μ*L of frozen-thawed semen from all concentrations of glycine were examined for total motility, motility kinematics, and progressive motility by a preheated glass slide and coverslip using 100× magnification. A minimum 400 spermatozoa from each sample were calculated under microscopic. Spermatozoa motility kinematics such as curvilinear velocity (VCL *μ*m/s), straight line velocity (VSL *μ*m/s), average-path velocity (VAP *μ*m/s), distance average path (DAP *μ*m), linear distance (DSL *μ*m), linearity (VAP/VCL) and straightness (VSL/VCL), and beat cross frequency (BCF Hz) were analyzed. The machine setting for selected CASA parameters was made using previous procedure [27]. The spermatozoa had <40% progressive motility which was considered as low motile sperms having a speed of less than 5 *μ*m/s. By contrast, if spermatozoa had >65% progressive motility, they were referred as highly motile sperms with a forward progression/speed of 25 *μ*m/s. But in our study, the post-thaw sperm motility was obtained from 33.46 to 49.41 which were considered as progressive motile sperms enabling to impregnate the ovum which falls in the range of previous studies [28, 29].

#### 2.3.2. DNA Integrity Percentage

DNA integrity was evaluated by using the acridine orange (AO) (Sigma, Aldrich, USA) solution of stain which was made from 10 mL stock and then added to one-liter distilled water and mixed and stored at 4°C temp in dark. A 40 mL of 0.1 M citric acid solution, 2.5 mL of 0.3 molar disodium phosphate. The pH of the solution was adjusted up to 2.5. A single drop of semen was put on standard glass slide, and then, smear was made and air dried, and the slide was fixed for 2 hrs in Carnoy's solution. A slide was stained with AO for three minutes and finally examined under phase contrast microscope (Olympus CX-41, Japan). A total of 250 spermatozoa per smear were estimated for DNA abnormalities [30].

#### 2.3.3. Mitochondrial Membrane Potential

A 50 *μ*L of frozen-thawed semen sample was diluted with 50 *μ*L tris-citric acid-fructose (TCF) and centrifuged at 300 g for five minutes. Spermatozoa pellet was added with TCF to make a volume up to 245 *μ*L, plus added with 5 mL Rhodamine (RH-123, Sigma Aldrich, USA), and incubated at room temperature for twenty minutes. A 50 *μ*L drop was placed on glass slide, and a coverslip was applied and examined under fluorescence microscope (48-0/550 nm excitation/barrier filter by using Olympus CX 41, Japan). At least 200 spermatozoa were observed for the presence of green fluorescence at midpiece and were considered to have normal intact mitochondrial membrane [31].

#### 2.3.4. Viability Percentage

The viability of spermatozoa was examined by using propidium iodide (PI) under florescent microscope. A 50 *μ*L tris-citric acid-fructose (TCF) was added to the 50 *μ*L of semen from each group concentration of glycine and centrifuged (300 g for five minutes) resulting in spermatozoa pellet. A volume of 2.5 *μ*L of PI was mixed to spermatozoa pellet after resuspending TCF to a volume of 47.5 *μ*L. Later on, the spermatozoa were stored at 37°C for five minutes. A total of at least 200 spermatozoa were calculated under the microscope to evaluate spermatozoa viability. Nonviable spermatozoa were noted in red color under the fluorescence microscope (Olympus CX-41, Japan) [32].

#### 2.3.5. Acrosome Integrity Percentage

Normal apical-ridge (NAR) solution consisting of 1% formal citrate (formaldehyde 37%, v/v Merck and 2.9%, w/v trisodium-citrate dehydrate, Merck, USA) was used for assessment of acrosomal integrity. A 500 *μ*L frozen-thawed semen was added with 50 *μ*L of 1% formal citrate formaldehyde and observed under phase contrast microscope (100×), and spermatozoa with viable intact acrosome had a sharp black crescent on their apical ridges [33].

#### 2.3.6. Plasma Membrane Integrity

The plasma membrane integrity (PMI) of spermatozoa was examined by using hypo-osmotic swelling test (HOST). A 50 *μ*L of semen sample was mixed with 500 *μ*L solution of HOS and placed for 30 min at 37°C in incubator. After incubation, 5 *μ*L semen droplets were examined under advance microscope (400×). A total of 100 spermatozoa were calculated for swelling in HOS solution. Spermatozoa swollen were recognized by coiling of spermatozoa tail impaired with plasma membrane [34].

#### 2.3.7. Post-Thaw Semen Total Antioxidant Capacity (T-AOC)

A total antioxidant capacity (TAC) colorimetric assay kits were used for measurement of a range of antioxidant macromolecules or protein antioxidants, and enzymes in a system can eradicate all types of reactive oxygen species and inhibit oxidative stress [35]. The entire level reflects the capacity of total antioxidant in the system. Numerous antioxidants in the body can diminish Fe3^+^ to Fe^2+^, and Fe^2+^ can form stable complexes with phenanthroline substances. The antioxidant capability (T-AOC) can be premeditated by measuring the absorbance at 520 nm. The data was computed through the following company protocol after obtaining the OD value (Elabscience T-AOC, colorimetric assay kit).

### 2.4. Statistical Design

Statistical analysis by one-way analysis of variance (ANOVA) and differences among treatment groups were determined by post hoc Duncan's multiple range test using SAS (version 9.1). Data was presented as mean ± SE. Differences were considered significant at *P* < 0.05.

## 3. Results

### 3.1. Influence of Glycine on Post-Thaw Motility Quality Parameters

#### 3.1.1. Spermatozoa Motility, Kinematics, and Velocity Distribution

The progressive fast motility post-thawed CASA parameters like total spermatozoa motility, progressive slow motility (%), and progressive fast motility (%) are shown in Table 2. Post-thawed total spermatozoa motility was significantly high (*P* < 0.05) in 10 mM glycine concentration (56.77 ± 2.59) as compared to other concentrations. At 15 mM concentration, the total spermatozoa motility was (46.97 ± 1.75) but lower than 10 mM followed by 5 mM (45.81 ± 0.80) and 20 mM (42.35 ± 1.09) concentration of glycine, respectively. However, the lowest total spermatozoa motility was recorded in control group (41.54 ± 0.68). The progressive linear motility (%), the progressive linear fast motility (%), and the progressive slow motility (%) were significantly higher (*P* < 0.05) in semen extender group containing 10 mM glycine concentration in comparison to control and other remaining glycine concentrations. Progressive motility (%) at 10 mM was 49.41 ± 2.12 followed by 5 mM (39.33 ± 1.08), 15 mM (38.30 ± 1.44), 20 mM (34.80 ± 1.36), and control (33.46 ± 1.78). The progressive fast motility (%) was recorded higher 27.80 ± 1.75 at 10 mM followed by 20.41 ± 1.71, 17.35 ± 1.62, and 16.67 ± 1.22 at 5 mM, 15 mM, and 20 mM glycine concentrations.

In current study, the curvilinear velocity (*μ*m/s) was higher at (*P* < 0.05) 10 mM that is 82.27 ± 3.27 followed by 69.6 ± 4.25, 64.83 ± 2.83, and 63.63 ± 2.01 at 20 mM, 15 mM, and 05 mM, respectively. The lowest curvilinear velocity (*μ*m/s) (54.48 ± 2.97) was recorded in control. The straight line velocity (*μ*m/s) was significantly high (*P* < 0.05) at 10 mM (30.40 ± 1.03) glycine concentration (27.66 ± 1.70) at 20 mM of glycine concentration followed by 26.13 ± 1.31 and 25.32 ± 3.00 at 5 mM and 15 mM concentrations, respectively.

The average path velocity (*μ*m/s) followed the same trend as it was higher (*P* < 0.05) at 10 mM (40.04 ± 1.02) glycine concentrations. The other glycine concentrations had lowered average path velocity (*μ*m/s), i.e., 33.06 ± 1.87, 32.20 ± 2.00, and 32.13 ± 1.51 at 20 mM, 15 mM, and 5 mM glycine concentrations, respectively. The control had lowered value of average path velocity (*μ*m/s) (27.6 ± 1.47) than other glycine concentrations. However, the value for linear distance (*μ*m/s) was recorded higher in 5 mM (9.50 ± 0.82) glycine concentration followed by 8.07 ± 0.85, 8.04 ± 0.38, and 7.43 ± 0.50 at 10 mM, 15 mM, and 20 mM, respectively. The control group has shown the lowest value, i.e., 7.38 ± 0.76 for linear distance (*μ*m/s).

The post-thawed CASA parameters like total velocity distribution values are shown in Table 3. The distance average path (*μ*m/s) was found significantly higher (12.22 ± 0.81) in 5 mM glycine concentration. The other values showed lower distance average path (*μ*m/s) that are 11.80 ± 0.77, 10.40 ± 0.55, and 9.94 ± 0.52 at 10 mM, 15 mM, and 20 mM glycine concentrations, respectively. The control group shows the lowest value (9.93 ± 0.75) for distance average path (*μ*m/s) as shown in Table 3. Beat cross frequency (Hz) is one of the other CASA parameters for spermatozoa. Beat cross frequency (Hz) is higher (8.80 ± 0.76) (*P* < 0.05) in semen extenders containing 10 mM glycine concentration in comparison to control and other glycine concentrations presented in Table 4. The other values for linearity (VSL/VCL) and straightness (VSL/VAP) were not found significantly correlated with each other in different glycine concentration.

#### 3.1.2. Post-Thawed Spermatozoa Quality Parameters

Post-thawed viability (%) was higher (51.08 ± 0.87) (*P* < 0.05) at 10 mM glycine concentration as compared to control and other glycine concentrations. It was followed by 5 mM concentration having 47.58 ± 0.86 viability%. The other glycine concentrations had 44.93 ± 0.46 and 41.65 ± 0.38 viability% for 15 mM and 20 mM, respectively. The control group had lower viability%, i.e., 44.22 ± 1.14, as compared to all other glycine concentrations as shown in Table 5. The plasma membrane integrity (PMI) percentage was also significantly higher (*P* < 0.05) at 10 mM (53.14 ± 0.41) glycine concentration in comparison to control and other glycine concentrations. The PMI% was 45.07 ± 0.61 at 5 mM followed by 43.92 ± 0.49 and 43.35 ± 0.58 at 20 mM and 15 mM, respectively. The control had lower value (43.28 ± 0.44) as compared to other glycine concentrations. The mitochondrial membrane potential was also significantly higher (50.72 ± 0.44), (*P* < 0.05) at 10 mM glycine concentration in comparison to control and other glycine concentrations. The mitochondrial membrane potential for other concentrations was 46.41 ± 0.94, 45.58 ± 0.61, and 44.93 ± 0.76 for 5 mM, 20 mM, and 15 mM, respectively. Post-thawed semen parameters viability percentage, plasma membrane integrity, and mitochondrial membrane potential of Achai bull semen are shown in Table 5.

However, acrosome (%) was significantly high (*P* < 0.05) at 10 mM (50.72 ± 0.21), followed by 5 mM (50.15 ± 0.57), 15 mM (50.08 ± 0.55), and 20 mM (48.72 ± 0.58) of glycine concentration as compared to control (48.43 ± 0.44). The DNA integrity was significantly high (*P* < 0.05) at 10 mM (98.93 ± 0.20) glycine concentration. At different glycine concentrations 5 mM, 15 mM, and 20 mM, the values for DNA integrity percentage were 98.15 ± 0.43, 98.01 ± 0.83, and 95.65 ± 0.76, respectively. Post-thawed DNA and acrosome integrity are presented in Table 6.

#### 3.1.3. Post-Thaw Total Antioxidant Capacity (T-AOC)

Post-thaw total antioxidant capacity (T-AOC) was significantly higher (*P* < 0.05) in samples having 10 mM (82.29 ± 1.19) of glycine concentration as compared to control and other concentrations. T-AOC was 67.28 ± 1.63, 75.55 ± 1.98, and 79.29 ± 0.68 at 5 mM, 15 mM, and 20 mM glycine concentrations, respectively. The T-AOC values are lower in control as compared to other glycine concentrations presented in post-thaw semen profile as shown in Table 6.

## 4. Discussion

This research was designed to investigate the effect of different concentrations of glycine on cryopreservation of Achai-bull semen. During the process of cryopreservation, half of the cells get damaged due to change in osmolality and oxidative stresses [36]. Oxidative stress in the semen occurs due to change in temperature in cryopreservation, resulting in irreparable injury to spermatozoa membrane and different organelles and changing in the antioxidant profile. These are some factors which lead to decreased spermatozoa motility, damage in spermatozoa membrane integrity, and ultimately lower fertility [37]. Spermatozoa plasma membrane is composed of large quantities of polyunsaturated fatty-acids (PUFA) which makes it vulnerable to oxidative stress [38, 39]. Glycine possesses antioxidant properties and shows scavenging effects against free radicals. Glycine showed significant role in the production of antioxidant enzymes that stimulates the protection system of spermatozoa against different oxidative stressors [40]. In current study, the optimal effect was observed at 10 mM of glycine concentration on post-thawed spermatozoa motility parameters.

Semen quality parameters were estimated by CASA which shows that glycine improved spermatozoa quality parameters and antioxidant capacity of cryopreserved semen. Post-thawed total spermatozoa motility was highly significant at 10 mM glycine concentration as compared to other glycine concentrations and control. Although progressive linear motility (%), progressive fast motility (%), and progressive slow motility (%) were higher at significant level in semen extender containing 10 mM glycine concentration in comparison to control and other glycine concentrations, in current study, the curvilinear velocity (*μ*m/s), the straight line velocity (*μ*m/s), and the average path velocity (*μ*m/s) were higher at (*P* < 0.05) 10 mM as compared to other glycine concentrations and control. However, the values of linear distance (*μ*m/s) and distance average path (*μ*m/s) were higher in 5 mM glycine concentrations as compared to other glycine concentrations and control. The current study findings are in agreement with [41, 42] in which they concluded that adding 25 mM glycine, glutamine, and 5 mM cysteine extender enhanced post-thawed motility, and improved plasma membrane and acrosome integrity of buffalo bull semen. In another study, Domosławska et al. [43] reported antioxidant capability of vitamin E, vitamin C, and its combined effect (vitamin E + C) on semen quality parameters, i.e., motility, percentage of live spermatozoa, percentage of abnormal spermatozoa, and acrosome intactness in the cryopreserved Bhadawari bull semen. They concluded that combined effect of paired vitamins has profound impact in protecting spermatozoa against production of reactive oxygen species (ROS) and cold shock in comparison to the only supplementation of vitamin E and vitamin C in the semen extender for cryopreservation.

Post-thawed viability (%), plasma membrane integrity, PMI percentage, and mitochondrial membrane potential (MMP) were significantly higher (*P* < 0.05) at 10 mM glycine concentration in comparison to control and other glycine concentrations. In addition, acrosome integrity (%) was significantly high (*P* < 0.05) at 10 mM (50.72 ± 0.21), followed by 5 mM, 15 mM, and 20 mM of glycine concentration and as compared to control group. The DNA integrity was found significant (*P* < 0.05) at 10 mM glycine concentration as compared to other glycine concentrations and control. The findings of this study are in line with Khalili et al. [44], who determined the effect of glycine and cysteine in different concentrations on numerous quality parameters of spermatozoa like motility, viability, acrosome integrity, and membrane integrity. The results indicate that the supplementation of 10 and 15 mM glycine and cysteine, respectively, in comparison to control extender significantly enhanced the motility, viability, and membrane integrity of cryopreserved spermatozoa, while the supplementation of increased quantity of amino acids up to 20 mM had a significant negative effect. Keeping in view this effect, addition of glycine and Cystine was recommended in extenders for cryopreservation of semen.

Post-thawed total antioxidant capacity (T-AOC) was higher (*P* < 0.05) in extender having 10 mM of glycine concentration in comparison to control and all other remaining concentrations. The T-AOC values for all other concentrations and control were lower than 10 mM glycine concentrations. These findings are in line with Shannon [45], who described the effect of diluents containing glycine and glycerol, on the fertility of diluted bovine semen. He concluded that the diluents containing glycine showed 3% increase in conception proving that glycine might improve the semen quality. These are also in line with the current findings in which pretreatment with alpha-lipoid acid supplementation reduced oxidative stress and improved semen quality [46]. The enhancement in spermatozoa antioxidant profile demonstrates the valuable addition of ALA in semen extender, motility kinematics, and velocity distribution. The previous research [47, 48] conducted on bovine has shown that significant enhancement in post-thawed motility was observed when semen samples were supplemented with 1 mM ALA in combination with 2 mM cysteine. Moreover, increase in the levels of ALA concentration decreased the spermatozoa motility parameters, and this was attributed to the change and lowering in semen pH, which was detrimental to spermatozoa resulting in immobility and death [49]. In our current research, results on best post-thaw semen parameters were obtained in semen containing 0.5 mM ALA, which is lowest concentration as compared to earlier study [47, 48].

## 5. Conclusion

It is concluded that addition of glycine at low level of 10 mM concentration along with vitamin E improved post-thaw total motility of Achai bull semen. The progressive total and progressive fast motility was also improved by the use of glycine @ 10 mM, and the supplementation of glycine coupled with vitamin E enhanced the total antioxidant capacity of cryopreserved semen, ultimately resulting in better conception rate.

## Figures and Tables

**Table 1:** Composition of semen extender.

Component	Quantity
Tris	3.07 gm
Citric acid	1.64 gm
Fructose	1.26 gm
Benzyl penicillin	1000 IU/mL
Streptomycin sulfate	100 *μ*g/mL
Glycerol	5%
Egg yolk	15%
Doubled-distilled water	Added up to the volume of 100 mL

**Table 2:** Effect of glycine semen extender on post-thaw CASA parameter (mobility and motility%) of Achai bull semen. Different superscripts represent the level of significance (*P* < 0.05) between the treatments and the control group. Different superscripts of the values in same row indicate significantly (*P* < 0.05) different among the concentrations.

Concentration of glycine (mM)	Total motility (%)	Progressive motility (%)	Progressive fast motility (%)	Progressive slow motility (%)
0	41.54 ± 0.68^c^	33.46 ± 1.78^c^	13.68 ± 1.60^d^	19.60 ± 0.76^ab^
5	45.81 ± 0.80^b^	45.81 ± 0.80^b^	20.41 ± 1.71^d^	18.34 ± 1.84^ab^
10	56.77 ± 2.59^a^	49.41 ± 2.12^a^	27.80 ± 1.75^a^	21.53 ± 1.80^a^
15	46.97 ± 1.75^b^	38.30 ± 1.44^b^	16.67 ± 1.22^c^	20.73 ± 1.24^a^
20	42.35 ± 1.09^c^	34.80 ± 1.36^c^	17.35 ± 1.62^c^	16.51 ± 1.63^b^

**Table 3:** Effect of glycine semen extender on post-thaw using CASA (velocity distribution) of Achai bull semen. In this table, different superscripts represent the level of significance (*P* < 0.05) between the treatments and the control group. Different superscripts of the values in same row show significant difference among groups (*P* < 0.05).

Concentration of glycine (mM)	Curvilinear velocity (*μ*m/s)	Straight line velocity (*μ*m/s)	Average path velocity (*μ*m/s)	Linear distance (*μ*m/s)
0	54.48 ± 2.97^c^	22.02 ± 1.48^c^	27.6 ± 1.47^d^	7.38 ± 0.76^b^
5	63.63 ± 2.01^b^	26.13 ± 1.31^b^	32.13 ± 1.51^c^	9.50 ± 0.82^a^
10	82.27 ± 3.27^a^	30.40 ± 1.03^a^	40.04 ± 1.02^a^	8.07 ± 0.85^b^
15	64.83 ± 2.83^b^	25.32 ± 3.00^b^	32.20 ± 2.00^c^	8.04 ± 0.38^ab^
20	69.6 ± 4.25^b^	27.66 ± 1.70^b^	33.06 ± 1.87^b^	7.43 ± 0.50^b^

**Table 4:** Effect of glycine as semen extender on post-thaw quality using CASA (kinematics) of Achai bull semen. In this table, different superscripts represent the level of significance (*P* < 0.05) between the treatments and control group. Different superscripts of the values in same row show significant difference among groups (*P* < 0.05).

Concentration of glycine (mM)	Distance average path (*μ*m/s)	Beat cross frequency (Hz)	Linearity (VSL/VCL)	Straightness (VSL/VAP)
0	9.93 ± 0.75^d^	6.62 ± 0.35^d^	0.41 ± 0.02^b^	0.80 ± 0.01^c^
5	12.22 ± 0.81^a^	8.18 ± 0.47^b^	0.41 ± 0.01^b^	0.81 ± 0.01^b^
10	11.80 ± 0.77^b^	8.80 ± 0.76^a^	0.38 ± 0.01^c^	0.77 ± 0.01^d^
15	10.40 ± 0.55^c^	7.51 ± 0.29^c^	0.43 ± 0.02^a^	0.81 ± 0.01^b^
20	9.94 ± 0.52^d^	6.95 ± 0.29^d^	0.43 ± 0.01^a^	0.82 ± 0.00^a^

**Table 5:** Effect of glycine extender on post-thaw semen parameter (viability%, plasma membrane integrity, mitochondrial membrane potential) of Achai bull semen. In this table, different superscripts represent the level of significance (*P* < 0.05) between the treatments and control group. Different superscripts of the values in same row show significant (*P* < 0.05) difference among groups.

Concentration of glycine (mM)	Viability%	PMI%	Mitochondrial membrane potential
0	44.22 ± 1.14^d^	43.28 ± 0.44^d^	44.70 ± 0.29^d^
5	47.58 ± 0.86^b^	45.07 ± 0.61^b^	46.41 ± 0.94^b^
10	51.08 ± 0.87^a^	53.14 ± 0.41^a^	50.72 ± 0.44^a^
15	44.93 ± 0.46^c^	43.35 ± 0.58^d^	44.93 ± 0.76^d^
20	41.65 ± 0.38^e^	43.92 ± 0.49^c^	45.58 ± 0.61^c^

**Table 6:** Effect of glycine in extender on post thaw semen parameter (acrosomal, DNA integrity and T-AOC) of Achai bull semen. In this table, different superscripts represent the level of significance (*P* < 0.05) between the treatments and control.

Concentration of glycine (mM)	Acrosome integrity%	DNA integrity%	Total antioxidant capacity (T-AOC)
0	48.43 ± 0.44^c^	96.33 ± 0.85^c^	33.26 ± 1.95^d^
5	50.15 ± 0.57^b^	98.15 ± 0.43^d^	67.28 ± 1.63^b^
10	50.72 ± 0.21^a^	98.93 ± 0.20^a^	82.29 ± 1.19^a^
15	50.08 ± 0.55^b^	98.01 ± 0.83^b^	75.55 ± 1.98^c^
20	48.72 ± 0.58^c^	95.65 ± 0.76^d^	79.29 ± 0.68^d^

## Data Availability

All data used in this study are included in this article. The primary data are available from the corresponding author on reasonable request.

## References

[1] Wing E. A. S. (2009). Government of Pakistan, FD. *Economic advisor’s wing, Islamabad*.

[2] Saleem M., Rahim I., Jalali S. (2013). Morphological characterization of Achai cattle in sedentary and transhumant systems in Pakistan. *Animal Genetic Resources*.

[3] Saleem M., Rahim I. U., Rueff H. (2012). Effect of management on reproductive performances of the Achai cattle in the Hindu Kush (northern Pakistan). *Tropical Animal Health and Production*.

[4] Kumar A., Prasad J. K., Srivastava N., Ghosh S. K. (2019). Strategies to minimize various stress-related freeze-thaw damages during conventional cryopreservation of mammalian spermatozoa. *Biopreservation and Biobanking*.

[5] O'Flaherty C., Vaisheva F., Hales B. F., Chan P., Robaire B. (2008). Characterization of sperm chromatin quality in testicular cancer and Hodgkin’s lymphoma patients prior to chemotherapy. *Human Reproduction*.

[6] Doshi S. B., Khullar K., Sharma R. K., Agarwal A. (2012). Role of reactive nitrogen species in male infertility. *Reproductive Biology and Endocrinology*.

[7] Agarwal A., Gupta S., Sharma R. K. (2005). Role of oxidative stress in female reproduction. *Reproductive Biology and Endocrinology*.

[8] Bucak M. N., Keskin N., Ili P. (2020). Decreasing glycerol content by co-supplementation of trehalose and taxifolin hydrate in ram semen extender: microscopic, oxidative stress, and gene expression analyses. *Cryobiology*.

[9] Zhong R.-Z., Zhou D.-W. (2013). Oxidative stress and role of natural plant derived antioxidants in animal reproduction. *Journal of Integrative Agriculture*.

[10] Marri V., Richner H. (2014). Differential effects of vitamins E and C and carotenoids on growth, resistance to oxidative stress, fledging success and plumage colouration in wild great tits. *The Journal of Experimental Biology*.

[11] Baumber J., Ball B. A., Gravance C. G., Medina V., Davies-Morel M. C. (2000). The effect of reactive oxygen species on equine sperm motility, viability, acrosomal integrity, mitochondrial membrane potential, and membrane lipid peroxidation. *Journal of Andrology*.

[12] Ugur M. R., Dinh T., Hitit M. (2020). Amino acids of seminal plasma associated with freezability of bull sperm. *Frontiers in Cell and Development Biology*.

[13] Wang W., Wu Z., Dai Z., Yang Y., Wang J., Wu G. (2013). Glycine metabolism in animals and humans: implications for nutrition and health. *Amino Acids*.

[14] Buranaamnuay K. (2020). Effect of different permeable cryoprotectants on the quality of cat epididymal spermatozoa. *Cryo Letters*.

[15] El-Sheshtawy R., El-Sisy G., El-Nattat W. (2008). Use of selected amino acids to improve buffalo bull semen cryopreservation. *Global Veterinaria*.

[16] Allai L., Benmoula A., Marciane da Silva M., Nasser B., el Amiri B. (2018). Supplementation of ram semen extender to improve seminal quality and fertility rate. *Animal Reproduction Science*.

[17] Soni Y., Talluri T. R., Kumar A., Ravi S. K., Mehta J. S., Tripathi B. N. (2019). Effects of different concentration and combinations of cryoprotectants on sperm quality, functional integrity in three Indian horse breeds. *Cryobiology*.

[18] Wasilewska-Sakowska K., Zasiadczyk Ł., Fraser L., Strzeżek J., Karpiesiuk K. (2019). Effect of post-thaw supplementation of fractionated seminal plasma on survival of boar spermatozoa. *Polish Journal of Veterinary Sciences*.

[19] Peña F. J., Johannisson A., Wallgren M., Rodriguez Martinez H. (2003). Antioxidant supplementation In Vitro improves boar sperm motility and mitochondrial membrane potential after cryopreservation of different fractions of the ejaculate. *Animal Reproduction Science*.

[20] Breininger E., Beorlegui N. B., O’Flaherty C. M., Beconi M. T. (2005). Alpha-tocopherol improves biochemical and dynamic parameters in cryopreserved boar semen. *Theriogenology*.

[21] Ayaz M., Ahmed A., Khan M. I., Yousaf M. S., Din B. U., Riaz A. (2020). Addition of alpha-lipoic acid in semen extender improves post-thaw antioxidant profile and semen quality of Achai (Bos indicus) cattle bulls. *JAPS: Journal of Animal & Plant Sciences*.

[22] Rehman Z. U., Samo M. U., Qureshi T. A. (2012). Studies on the freezability of Kundhi buffalo bull semen. *Journal of Animal and Plant Sciences*.

[23] Aalseth E. P., Saacke R. G. (1987). Alteration of the anterior acrosome of motile bovine spermatozoa by fructose and hydrogen ion concentration. *Journal of Reproduction and Fertility*.

[24] Susilowati S., Sardjito T., Mustofa I., Widodo O. S., Kurnijasanti R. (2021). Effect of green tea extract in extender of simmental bull semen on pregnancy rate of recipients. *Anim Biosci*.

[25] Hu J. H., Zhao X. L., Tian W. Q., Zan L. S., Li Q. W. (2011). Effects of vitamin E supplementation in the extender on frozen-thawed bovine semen preservation. *Animal*.

[26] PARC/JICA (1986). *Manual on artificial insemination in water buffaloes and cattles*.

[27] Chapin R. E., Filler R. S., Gulati D. (1992). Methods for assessing rat sperm motility. *Reproductive Toxicology*.

[28] Gangwar C., Saxena A., Patel A. (2018). Effect of reduced glutathione supplementation on cryopreservation induced sperm cryoinjuries in Murrah bull semen. *Animal Reproduction Science*.

[29] Shenkute Goshme T. A., Besufekad S. (2021). Evaluation of motility and morphology of frozen bull semen under different thawing methods used for artificial insemination in North Shewa zone, Ethiopia. *Heliyon*.

[30] Tejada R. I., Mitchell J. C., Norman A., Marik J. J., Friedman S. (1984). A test for the practical evaluation of male fertility by acridine orange (AO) fluorescence. *Fertility and Sterility*.

[31] Dodaran H. V., Zhandi M., Sharafi M. (2015). Effect of ethanol induced mild stress on post-thawed bull sperm quality. *Cryobiology*.

[32] Aquila S., Giordano F., Guido C., Rago V., Carpino A. (2011). Nitric oxide involvement in the acrosome reaction triggered by leptin in pig sperm. *Reproductive Biology and Endocrinology*.

[33] Rasul Z., Ahmad N., Anzar M. (2001). Changes in motion characteristics, plasma membrane integrity, and acrosome morphology during cryopreservation of buffalo spermatozoa. *Journal of Andrology*.

[34] Ramu S., Jeyendran R. S. (2013). The hypo-osmotic swelling test for evaluation of sperm membrane integrity. *Methods in Molecular Biology*.

[35] Agarwal A., Roychoudhury S., Bjugstad K. B., Cho C. L. (2016). Oxidation-reduction potential of semen: what is its role in the treatment of male infertility?. *Therapeutic Advances in Urology*.

[36] Watson P. F. (2000). The causes of reduced fertility with cryopreserved semen. *Animal Reproduction Science*.

[37] Contreras M. J., Treulen F., Arias M. E. (2020). Cryopreservation of stallion semen: effect of adding antioxidants to the freezing medium on sperm physiology. *Reproduction in Domestic Animals*.

[38] Alonge S., Melandri M., Leoci R., Lacalandra G., Caira M., Aiudi G. (2019). The effect of dietary supplementation of vitamin e, selenium, zinc, folic acid, and N-3 polyunsaturated fatty acids on sperm motility and membrane properties in dogs. *Animals*.

[39] Alvarez J. G., Storey B. T. (1995). Differential incorporation of fatty acids into and peroxidative loss of fatty acids from phospholipids of human spermatozoa. *Molecular Reproduction and Development*.

[40] Packer L., Kraemer K., Rimbach G. (2001). Molecular aspects of lipoic acid in the prevention of diabetes complications. *Nutrition*.

[41] Shakouri N., Soleimanzadeh A., Rakhshanpour A., Bucak M. N. (2021). Antioxidant Effects of Supplementation of 3,4-Dihydroxyphenyl Glycol on Sperm Parameters and Oxidative Markers Following Cryopreservation in Canine Semen. *Reproduction in Domestic Animals*.

[42] Kutluyer F., Kocabas M. (2016). Use of selected amino acids to improve buffalo bull semen cryopreservation. *Austin. Biol.*.

[43] Domosławska A., Zdunczyk S., Franczyk M., Kankofer M., Janowski T. (2018). Selenium and vitamin E supplementation enhances the antioxidant status of spermatozoa and improves semen quality in male dogs with lowered fertility. *Andrologia*.

[44] Khalili B., Jafaroghli M., Farshad A., Paresh-Khiavi M. (2010). The effects of different concentrations of glycine and cysteine on the freezability of moghani ram spermatozoa. *Asian-Australasian Journal of Animal Sciences*.

[45] Shannon P. (1964). The effect of diluents containing glycine, and glycine and glycerol, on the fertility of diluted bovine semen. *New Zealand Journal of Agricultural Research*.

[46] Taherian S. S., Khayamabed R., Tavalaee M., Nasr-Esfahani M. H. (2019). Alpha-lipoic acid minimises reactive oxygen species-induced damages during sperm processing. *Andrologia*.

[47] Bucak M. N., Ataman M. B., Başpınar N. (2015). Lycopene and resveratrol improve post-thaw bull sperm parameters: sperm motility, mitochondrial activity and DNA integrity. *Andrologia*.

[48] Bucak M. N., Ateşşahin A., Yüce A. (2008). Effect of anti-oxidants and oxidative stress parameters on ram semen after the freeze-thawing process. *Small Ruminant Research*.

[49] Olmsted S. S., Dubin N. H., Cone R. A., Moench T. R. (2000). The rate at which human sperm are immobilized and killed by mild acidity. *Fertility and Sterility*.

